# Sports Medical Image Modeling of Injury Prevention in Dance Learning and Sports Training

This article has been retracted.

**DOI:** 10.1155/2022/7027007

**Published:** 2022-07-27

**Authors:** Renying Fei

**Affiliations:** Liupanshui Normal University, Liupanshui, Guizhou 553004, China

## Abstract

In order to effectively prevent injuries in dance learning and sports training, this paper proposes a method based on sports medical image modeling. This method solves the problem of injury prevention in dance learning by studying the association analysis algorithm, medical image information system, and CT technology and analyzing the role of data mining technology in the medical image information system. The experimental results show that the average prediction error of CT and US is about 5%, which can be considered that the model can predict accurately. The error of MR is as high as 28.2%, and the prediction is relatively inaccurate. *Conclusion*. the model can effectively prevent the injury in training.

## 1. Introduction

In order to interpret the dance performance perfectly during the training process, dancers often need to do some difficult movements, which will cause dance sports injuries. The sports injury caused by dance training is often complex; such sports injuries are usually associated with dance training. Dance sports injuries may require rehabilitation at least or may lead to the end of dance sports career [1]. Many excellent dancers and dancers have to say goodbye to their dance career and give up their favorite dance career because of sports injury. It can be said that dance sports injury has become a problem that many dancers have to face. Therefore, it is very important to prevent injuries in the process of dance learning.

Medical imaging is an equipment-dependent discipline. Medical imaging equipment, especially CT and MR equipment, is driven by the most rapidly developing cutting-edge technology in natural science and is developing at a veritable speed [2–4]. At each stage of the development of medical imaging, it will have an important and sometimes epoch-making impact on other clinical disciplines closely related to it. At present, the development of medical imaging represented by the development of CT and MR technology is at such a stage. Among them, data mining technology plays an important role in medical imaging [5]. Data mining technology is a process of extracting hidden, unknown, but potentially useful information and knowledge from a large number of incomplete, noisy, fuzzy, and random practical application data. This process generally consists of the data preparation stage, data mining stage, and result expression and interpretation stage (see Figure 1). The data preparation stage can be further divided into data integration, data selection, and data preprocessing; The mining operation stage includes determining the goal of data mining, selecting appropriate tools, mining knowledge, and verifying the discovered knowledge. The task of the result expression and interpretation stage requires not only expressing the results but also filtering the information. If the results cannot satisfy the decision-maker, the above data mining process should be repeated.

Based on this, through the analysis of the injuries in dance training, and through the prevention of medical imaging technology, we can effectively prevent the injuries of dancers in the training process.

## 2. Literature Review

Dance sports injury refers to the emergency changes and changes in physiological and biochemical indicators of the dancer's body tissues or body structures and organs caused by multiple factors in the process of dance performance or dance training. These changes mainly occur in the basic motor system of dancers and also have adverse effects on the nervous system and vascular system. In order to present the most perfect side to the audience, dancers often carry out arduous training “day after day, year after year.” Such training often exceeds the physical limit, and long-term high-intensity training causes sports injuries to dancers. According to the research and analysis, the training injuries of dancers are usually caused by the following three reasons:

1. Insufficient preparation activities
2. Lack of tacit cooperation when two people cooperate
3. Low physical and psychological quality

In view of the reasons, it can effectively prevent serious injuries caused by dancers in the training process.

1998 is another epoch-making mark in the development of CT technology [6]. In this year, several major CT equipment manufacturers simultaneously launched four layer acquisition spiral CT (multislice spiral CT), and its principle has been introduced in other literatures [7]. Taking this as a starting point, the 8-layer spiral CT was launched in 2000. In 2001, the 16-slice spiral CT was introduced, and 2-slice, 6-slice, and 10-slice spiral CT with similar principle were also developed. Improved electron beam CT was introduced in 2002 [8].

The key breakthrough of multislice spiral CT is the use of a multirow wide body detector instead of single-row detector of the single-slice spiral CT [9]. By controlling the switch of the information channel of each detector column, the reconstructed images with 4 as the cardinal number and different layer thicknesses can be obtained. The detector width of the thinnest column in the multicolumn detector determines the thinnest acquisition layer thickness, i.e., *z*-axis resolution. For example, in the current detector design, the width of the thinnest column detector is 0.5 mm (Toshiba), 0.625 mm (GE), and 0.75 mm (Siemens and Philips), which is the thinnest layer thickness that can be collected by each equipment. The setting of the thinnest layer thickness is not random. It is closely related to several main performance parameters, namely, cone-shaped X-ray harness reconstruction mathematics, scanning speed, X-ray dose, computer performance, and voxel isotropy, which is highly valued in clinical applications [10–12].

Data mining technology is a process of extracting hidden, unknown, but potentially useful information and knowledge from a large number of incomplete, noisy, fuzzy, and random practical application data. This process generally consists of the data preparation stage, data mining stage, and result expression and interpretation stage. The data preparation stage can be further divided into data integration, data selection, and data preprocessing. The mining operation stage includes determining the goal of data mining, selecting appropriate tools, mining knowledge, and verifying the discovered knowledge. The task of the result expression and interpretation stage requires not only expressing the results but also filtering the information. If the results cannot satisfy the decision-maker, the above data mining process should be repeated. Data mining generally relies on professional tools. Common data mining technologies mainly include association rule analysis, artificial neural network, decision tree analysis, time series analysis, cluster analysis, etc. [13]. Focus on the application of association rule analysis and time series analysis in the medical image information system. With the development of medical informatization, more and more hospitals begin to popularize the application of the medical image information system, which is mainly composed of the medical image information system (RIS) and medical image archiving and transmission system (PACS) [14]. RIS is mainly responsible for examination registration, examination photography, report editing, review and follow-up, department management, and other functions, while PACS is mainly responsible for the acquisition, transmission, storage, display, and management of medical images. Over the years since the implementation of RIS/PACS in a class III hospital, the inspection records have reached more than 1 million, and the image records have reached more than 5 million. The massive data accumulated in the database provides a good foundation for data mining and utilization.

Based on the above research, this paper makes an in-depth discussion and research on the sports medical impact modeling of injury prevention in dance learning and sports training. Through the research of the association analysis algorithm, medical impact information system, and CT technology, data mining technology is applied to medical imaging technology, and finally, an effective prevention of dance training injury is achieved.

## 3. Research Methods

### 3.1. Correlation Analysis of Inspection Items

#### 3.1.1. Association Rule Algorithm

Association rules are used to filter out the frequency relationship of data item sets in the transaction database from a given set of data items and the transaction database (each transaction is a collection of data items) and to find valuable correlation between data item sets in a large amount of data. When mining association rules, various events in the database data must be taken as data items, and multiple data items form an itemset of a specific thing [15]. For example, in the medical image database, for the event of patient visit, each examination item in the process of visit constitutes its data item set. Microsoft association rule algorithm belongs to the Apriori rule algorithm series, which can be divided into two steps: one is to find all frequent itemsets whose support is greater than or equal to the predefined minimum support threshold; the other is to generate strong association rules that meet the minimum confidence from the frequent itemsets.

#### 3.1.2. Data Preparation

Due to the lack of necessary data verification during the use, maintenance, and migration of data for many years, coupled with the gradual launch of the software function module of the image information system, and the human error of the staff when entering the data, the data may be repeated, missing, incomplete, and wrong. Therefore, in order to ensure the quality of data, it is necessary to process the data.

The EISStudies (check information table) and EISService (item information sheet) in the RIS database of a hospital record the information about the examination items of patients in the hospital since 2005, from which the basic attributes of patients (number, name, gender, date of birth, etc.), patient types (physical examination, outpatient, emergency, inpatient), and examination items (number, name, type, etc.) are extracted to establish a new table. Because the original entry of inspection items is not standardized, the same inspection item has different numbers and names [16]. For example, (X-ray (digital) chest film (positive position) CR) and (X-ray (digital) chest film Cr (positive position)) are the same inspection item. In order not to affect the analysis results, the inspection items need to be uniformly standardized.

#### 3.1.3. Frequent Itemsets and Association Rules

The primary task of the association rule algorithm is to mine frequent itemsets. Due to the large number of patient examination items, in order to obtain useful itemsets and rules and reduce model processing time, the minimum support parameter is set to 0.03; that is, only itemsets with a frequency of not less than 3% are selected to generate association rules [17, 18].  Figure 2 shows the generation process of frequent itemsets.

According to the generation process of the above frequent itemsets, the model generates association rules (see Table 1), where confidence refers to the probability of the occurrence of result B when condition A occurs, importance refers to the logarithm of the ratio of the occurrence probability of the result when the condition is true to the occurrence probability of the result when the condition is not true, and the importance score is greater than zero, indicating that the rule is meaningful, and the greater the score, the more significant the rule is. It can be seen from Table 1 that in the physical examination items, the probability of color ultrasound B (kidney, ureter, bladder, prostate) and color ultrasound A (liver, gallbladder, spleen, pancreas) is 98.2%, and the importance score of the rule is 1.157. Among inpatients, the probability of taking chest DR at the same time of US project of the left and right lower limb deep vein was 73.1%, and the importance score of this rule was 2.867. It can be found that the patients whose type is physical examination have high confidence, which is consistent with the fact that the physical examination patients will do some combination packages of examination items. Because of the uncertainty of the examination items of outpatient and emergency patients, the confidence of the rules is generally not as high as that of the physical examination.

Through association rule analysis, we can find the association degree of the inspection items during the patient's visit. If we further combine the patient's disease type, it can provide a basis for the hospital's clinical path management.

### 3.2. Forecast of Equipment Inspection Quantity

#### 3.2.1. Timing Algorithm

The Microsoft time series algorithm encapsulates two different computer learning algorithms. The first algorithm is the automatic regression tree (ARTxp) using cross-prediction, and the second algorithm is automatic regression (ARIMA) integrated with moving average. The Microsoft time series algorithm combines the advantages of the two algorithms by default to achieve the optimal prediction results [19].

#### 3.2.2. Establishment and Verification of Time Series Model

The modern imaging department has a large number of digital imaging equipment, such as CT, MR, CR, DR, and DF. It extracts and collects the monthly inspection quantity of each equipment type from the original eisservice in the RIS/PACS database and designs the monthly inspection quantity of equipment to establish the time series model. Since the data in the new table has been processed, there is no missing value, the data is summarized and recorded on a monthly basis, and the sequence cycle is set to 12.  Figure 3 is the flow chart of the timing model.

#### 3.2.3. Comprehensive Forecast

In statistics, multiple index systems are generally used for comprehensive prediction to improve the prediction accuracy of inspection volume [20]. Here, the examination volume in 2021 is comprehensively predicted according to the two index systems of the patient type and equipment type. Since the inspection volume prediction of the two indicator systems adopts the time series algorithm, now assuming that the importance of the indicator system is the same, the equal weight average method can be used to determine that the weight is 0.5.

(1) $$\begin{array}{c} Q_{1}=Q\left(\text{physical examination}\right)+Q\left(\text{hospitalization}\right)+Q\left(\text{emergency treatment}\right)+Q\left(\text{outpatient Department}\right), \end{array}$$

(2) $$\begin{array}{c} Q_{2}=Q_{\text{CT}}+Q_{\text{US}}+Q_{\text{CR}}+\cdots +Q, \end{array}$$

(3) $$\begin{array}{c} Q=0.5Q_{1}+0.5Q_{2}, \end{array}$$

where *Q* is the target predicted total examination volume, is the predicted total examination volume by patient type, and is the predicted total examination measurement by device type. After the total inspection quantity is obtained according to equation (3), the inspection quantity of each equipment type can be obtained according to the following equation:

(4) $$\begin{array}{c} Q_{\text{CT}}^{\prime }=Q_{\text{CT}}*\frac{Q}{Q_{2}}. \end{array}$$

After the comprehensive prediction model is determined, the time series model is used to predict the monthly examination volume of the imaging department in 2021 according to the patient type and equipment type index system. Due to the abrupt change of the MR examination volume in 2020, the direct prediction error according to the time series is large. Now, according to the historical data, the average growth rate of MR in recent years is calculated to be about 3.5%, and the growth rate has a trend of increasing year by year. After comprehensive consideration, 4% is added to the actual value in 2020 as the prediction result of the MR examination type in 2021.

After the total inspection amount of each equipment type is obtained, the total inspection amount in 2021 can be obtained according to equation (3), and then, the inspection amount of each equipment inspection type can be calculated according to equation (4).  Table 2 shows the predicted values of the inspection volume of each equipment type in 2021, the historical data from 2018 to 2020, and the growth of various inspection volumes in 2021. Based on this prediction result, the decision-makers can know the department equipment inspection volume in 2021 in advance, make the allocation of equipment and personnel in advance, and improve the decision-making management level. For example, in view of the high growth rate of CT in 2021, new CT equipment has been considered to actively respond to the growth of examination business to improve the quality of medical services [21].

### 3.3. CT Detector

The design of CT detector can specify the size of the pixel and matrix. When the earliest layer acquisition and display method is applied, the layer thickness only involves the distortion caused by “partial volume effect.” When using multislice spiral CT to display reconstructed images, it involves not only the concept of pixel and matrix but also the concept of voxel. The concept that pixels are “areas” is two-dimensional. “Voxel” is the concept of “volume,” which is three-dimensional, that is, length, width, and height. Where “length” and “width” are two-dimensional parameters of “pixels,” “height” is determined by the acquisition layer thickness. When the acquisition layer thickness is the same as “length” and “width,” the voxel is “isotropic”; otherwise, it is “anisotropic.” When using isotropic voxel data for reconstruction, the reconstructed image will not be distorted. If voxel data is anisotropic, the reconstructed image will be distorted to varying degrees.

In fact, in order to achieve isotropic voxel acquisition, it is necessary to select an appropriate field of view (FOV). When the data is collected with the quadratic matrix of 512, the design of a company needs to use 32 cm FOV to obtain 0.625 cubic mm isotropic voxels. The design of a company needs to adopt 38 cm FOV to obtain 0.75-cubic-millimeter isotropic voxels. The design of a company needs to select 25 cm FOV to obtain 0.5-cubic-millimeter isotropic voxels.

In addition to the acquisition method, this type of design also involves problems such as the high scanning dose, the need for new reconstruction algorithms, the need to greatly improve the computer capacity due to the large increase in the amount of data, and the cost and design of the flat panel detector itself (for example, the flat panel detector can only be placed horizontally, not in an arc) which need to be further solved.

## 4. Results and Discussion

Table 3 lists the actual value, predicted value, and relative error of each equipment type in 2020. It can be seen from the table that the average prediction error of CT and US is about 5%, so it can be considered that the model can predict more accurately. The error of MR is as high as 28.2%. The reason is that there is a sudden change in the inspection volume of MR from February to March 2020, which is much larger than in previous years. After in-depth understanding, it is the newly added inspection items in the hospital MR room after external training which lead to a significant increase in business volume and a large error in the time series prediction results. Therefore, it is appropriate to use this time series to predict CT and US volume, while other methods must be used to predict MR volume.  Figure 4 shows the line chart of relative error of each equipment.

It can be seen from Table 3 that the average prediction error of CT and US is about 5%, so it can be considered that the model can predict more accurately. The error of MR is as high as 28.2%, and the data mining technology is used to process the massive data accumulated in the application of the medical imaging information system (RIS/PACS) in a hospital for several years [22]. The association rule algorithm is mainly used to conduct association analysis on patient examination items, which provides a reference for hospital clinical path management, provides a certain technical basis for injury prediction in dance training, and effectively improves the prediction rate.

## 5. Conclusion

This paper studies the research of sports medical image modeling for injury prevention in dance learning and sports training, through the research of association analysis algorithm, medical image information system, and CT technology. This paper also analyzes the role of data mining technology in the medical image information system to solve the problem of injury prevention in dance learning. The experimental results show that the average prediction error of CT and US is about 5%, which can be considered that the model can predict accurately.

## Figures and Tables

**Figure 1:** Data mining process.

**Figure 2:** Generation process of frequent itemsets.

**Figure 3:** Flow chart of time series model.

**Figure 4:** Broken line statistics of relative errors of CT and US.

**Table 1:** Association rules.

Patient type	Generated association rules	Confidence (%)	Importance
Physical examination	Color ultrasound B (kidney, ureter, bladder, prostate)→color ultrasound A (liver, gallbladder, spleen, pancreas)	98.2	1.157
Hospitalization	Left and right lower limb deep vein US→chest DR	73.1	2.867
Emergency treatment	CR of limbs, plain scan of liver, gallbladder, spleen and pancreas→plain scan of head CT	66.4	1.512
Outpatient department	Chest DR, double arm ureter bladder prostate→liver, gallbladder, spleen, and pancreas	73.2	1.101

**Table 2:** Forecast of inspection volume of each equipment type in 2021.

	2018	2019	2020	2021	Forecast growth rate in 2021
CT	49391	60161	65705	71822	8.52%
US	157132	166843	178529	186691	4.37%
CR	26624	21708	22358	23429	4.57%
DR	44505	55208	55854	58588	4.67%
MR	15590	15831	22118	28852	4.00%

**Table 3:** Comparison of actual and predicted values of inspection quantities of various equipment types in 2020.

	CT			US			MR		
	Actual value	Estimate	Relative error	Actual value	Estimate	Relative error	Actual value	Estimate	Relative error
202001	4704	5020	0.0671	10946	12305	0.1239	1134	1189	0.0485
202002	4598	5112	0.1117	9732	11225	0.1534	1190	1043	0.1235
202003	5642	5518	0.0219	13757	14110	0.0256	1955	1424	0.2716
202004	5617	5678	0.0108	14338	14288	0.0034	1872	1388	0.2585
202005	5876	5772	0.0176	16591	15403	0.0716	1991	1365	0.3144
202006	5563	5782	0.0393	17100	15743	0.0793	2027	1436	0.2916
202007	5634	5748	0.0202	17409	17298	0.0063	2040	1427	0.3005
202008	5983	5864	0.0196	17314	16281	0.0596	2105	1155	0.4513
202009	5249	5897	0.1234	15988	14778	0.0756	1868	1335	0.2853
202010	5763	5991	0.0396	14772	14197	0.0389	2079	1336	0.3574
202011	5609	5841	0.0413	16180	15051	0.0697	2067	1252	0.3943
202012	5467	5972	0.0924	14400	14392	0.0005	1790	1276	0.2874
Average error	—	—	0.0504	—	—	0.0590	—	—	0.2820

## Data Availability

The data used to support the findings of this study are available from the corresponding author upon request.
